# Identification of Prognostic Biomarkers of Cutaneous Melanoma Based on Analysis of Tumor Mutation Burden

**DOI:** 10.1155/2020/8836493

**Published:** 2020-11-16

**Authors:** Jiaqiong Lin, Yan Lin, Zena Huang, Xiaoyong Li

**Affiliations:** ^1^Department of Medical Genetics, School of Basic Medical Sciences, Southern Medical University, Guangzhou, China; ^2^Department of Nephrology, Third Affiliated Hospital, Guangzhou Medical University, Guangzhou, China; ^3^Department of General Medicine, Guangdong Provincial People's Hospital, Guangdong Academy of Medical Sciences, Guangzhou, China; ^4^Department of General Surgery, Third Affiliated Hospital of Guangzhou Medical University, Guangzhou, China

## Abstract

**Background:**

Immunotherapy offers a novel approach for the treatment of cutaneous melanoma, but the clinical efficiency varies for individual patients. In consideration of the high cost and adverse effects of immunotherapy, it is essential to explore the predictive biomarkers of outcomes. Recently, the tumor mutation burden (TMB) has been proposed as a predictive prognosticator of the immune response.

**Method:**

RNA-seq and somatic mutation datasets of 472 cutaneous melanoma patients were downloaded from The Cancer Genome Atlas (TCGA) database to analyze mutation type and TMB. Differently expressed genes (DEGs) were identified for functional analysis. TMB-related signatures were identified via LASSO and multivariate Cox regression analysis. The association between mutants of signatures and immune cells was evaluated from the TIMER database. Furthermore, the Wilcox test was applied to assess the difference in immune infiltration calculated by the CIBERSORT algorithm in risk groupings.

**Results:**

C>T substitutions and TTN were the most common SNV and mutated gene, respectively. Patients with low TMB presented poor prognosis. DEGs were mainly implicated in skin development, cell cycle, DNA replication, and immune-associated crosstalk pathways. Furthermore, a prognostic model consisting of eight TMB-related genes was developed, which was found to be an independent risk factor for treatment outcome. The mutational status of eight TMB-related genes was associated with a low level of immune infiltration. In addition, the immune infiltrates of CD4+ and CD8+ T cells, NK cells, and M1 macrophages were higher in the low-risk group, while those of M0 and M2 macrophages were higher in the high-risk group.

**Conclusion:**

Our study demonstrated that a higher TMB was associated with favorable survival outcome in cutaneous melanoma. Moreover, a close association between prognostic model and immune infiltration was identified, providing a new potential target for immunotherapy.

## 1. Introduction

Cutaneous melanoma, characterized by high aggressiveness and poor prognosis, is well known as a common malignant neoplasm of the skin having the highest mortality rates [1, 2]. It is classified into different subtypes, including the lentigo malignant type, the superficial spreading type, and the nodular type based on clinical and histological characteristics [3]. Cutaneous melanoma originates from melanocytes, and its incidence has increased rapidly in recent years, causing serious problems to public health [4, 5]. When in the advanced stages, approximately 8% to 46% of patients develop brain metastasis [6]. Of note, in patients with metastasis, the 5-year survival rate dramatically declines to 10% [7, 8]. The therapeutic approaches vary considerably depending on the different tumor stages. Surgical resection remains a major treatment approach for the early stage of cutaneous melanoma. Combination with chemotherapy, radiotherapy, and targeted therapy after surgical intervention is required for most patients in advanced stages [9]. However, the treatment efficacy remains limited and the prognosis is poor for patients in advanced stages.

In recent years, immunotherapy, including CAR T cell therapy, monoclonal antibodies, vaccine, and immune checkpoint inhibitors (ICIs) has developed considerably and has established new perspectives for the treatment of these malignant neoplasms [10–12]. Notably, ICIs targeting the cytotoxic T-lymphocyte antigen 4 (CTLA-4), programmed death-ligand 1 (PD-L1), and programmed cell death receptor 1 (PD-1) bring a great promise for the treatment of patients with cutaneous melanoma [13, 14]. Nevertheless, effective biomarkers able to discriminate populations who would benefit most from the treatment of ICIs are still lacking. The drugs of ICIs are expensive, and patients benefit from each immunotherapeutic intervention differently, which raises difficulties in defining therapy. Hence, it is of great significance to be able to effectively discriminate those patients who may benefit from immunotherapy.

With the rapid development of sequencing technology and the growing understanding of tumorigenesis, precision-targeted therapy is emerging as a promising anticancer approach. Thanks to the public data repositories such as The Cancer Genome Atlas (TCGA) database; this abundant publicly available source of tumor data provides a valuable foundation for in-depth investigations. Several studies have demonstrated that the tumor mutation burden (TMB) is closely associated with immunotherapy outcomes in multiple cancer types and is emerging as a predictive biomarker for the response of immunotherapy [15–17]. The definition attributed to TMB is the total number of somatic mutations including base substitutions, deletions, and insertions detected in per one million bases [18]. The degree of TMB is possibly associated with multiple factors, such as microsatellite instability and environmental damage [19]. Mutations in driver genes could promote oncogenesis. Conversely, a large number of somatic mutations may produce a vast amount of neoantigens, serving as targets of activated immune cells [20]. Hence, the accumulation of somatic mutations in cancer has resulted in increased TMB and neoantigens, which can be recognized and attacked by the immune system [21]. Patients with higher TMB manifested a favorable response to immunotherapy [22]. In non-small-cell lung cancer (NSCLC), the TMB was identified as an effective predictor of response to treatment of ICIs [23]. In addition, Thomas et al. demonstrated that TMB played a crucial role in immune-mediated survival in patients with breast cancer [24]. Furthermore, it has been demonstrated that the role of TMB in the immune response and in immune infiltration varies depending on the tumor type [25]. A limited number of studies have investigated the relationship between TMB and prognostic prediction in cutaneous melanoma. Therefore, we conducted our present study to explore the potential role of TMB in cutaneous melanoma using public data resources.

## 2. Method

### 2.1. Data Collection

Somatic mutation datasets were downloaded from the TCGA database (https://portal.gdc.cancer.gov). Of these, the profiles processed by the VarScan software were chosen for further analysis and visualization using the “maftools” R package. In addition, transcriptome data including HTSeq-Counts and clinical data such as survival time and survival status, as well as other clinical futures of 472 samples with cutaneous melanoma including 1 normal sample and 471 tumor samples, were also obtained from the TCGA database. Samples with missing follow-up information were excluded; thus, a total of 460 samples were investigated in the study.

### 2.2. TMB Calculation

TMB, the total number of mutations per megabyte, was calculated by dividing the total number of variants by the overall size of human exons (38 Mb). Next, patients were stratified into low and high TMB groups according to the median value. The Kaplan-Meier analysis was employed to evaluate the survival function between the two groups. Furthermore, the relationship between the TMB levels and clinical characteristics was compared by the Wilcox test or Kruskal-Wallis test depending on the number of groups for comparison.

### 2.3. Identification and Functional Analysis of Differentially Expressed Genes

The DEG-seq2 R package was used to identify the differentially expressed genes (DEGs) between the low and high TMB groups, with ∣log2FC | >2 and FDR < 0.05 considered as threshold values. The volcano plot of genes was drawn using the R package with upregulated DEGs marked in red and downregulated DEGs in blue. Subsequently, the GO functional analysis of 403 DEGs and the gene set enrichment analysis (GSEA) of all genes were carried out via R packages including clusterProfiler, org.Hs.eg.db and ggplot2 [26].

### 2.4. Development and Assessment of the TMB-Related Prognostic Model

The prognosis-related DEGs extracted from a combined univariate Cox and Kaplan-Meier analysis were selected for the construction of the prognostic model utilizing the Lasso-penalized Cox regression analysis and multivariate Cox regression. The risk scores were calculated as follows: Riskscores = expressionofTGM3 × (0.0129) + expression of PROKR1 × (0.4339) + expression of CRABP2 × (0.0014) + expression of CHI3L1 × (−0.0024) + expression of PAEP × (0.0002) + expression of KLRK1 × (−0.7398) + expression of SLC32A1 × (−15.5098) + expression of SPRR2F × (0.0366). The distribution of the survival status of patients and TMB-related genes in the low- and high-risk score groupings was visualized using the R package. In addition, the Kaplan-Meier analysis was employed to compare the overall survival (OS) of each of the two groups. Univariate and multivariate Cox regression analyses were carried out to determine the independent prognostic factors for cutaneous melanoma. *p* < 0.05 indicated statistical significance. The Receiver Operating Characteristic (ROC) curve was employed to evaluate the performance of the prognostic model. Furthermore, a nomogram was established to predict the progression risk of cutaneous melanoma.

### 2.5. TIMER Database and Estimation of Immune Infiltration

The association between immune infiltration levels and mutation types of the prognostic genes was investigated via the TIMER database (https://cistrome.shinyapps.io/timer/). Significance testing utilizing the Wilcox test was employed to evaluate the immune infiltration levels in different mutation types. In addition, the CIBERSORT algorithm was conducted to evaluate the immune infarction in patients with cutaneous melanoma. The Wilcox test was performed to determine different immune infiltration levels between the low- and high-risk groups, and the results were visualized by violin plots.

### 2.6. Statistical Analysis

All analyses were performed by R version 3.6.3 and the corresponding packages. The Kaplan-Meier analysis was employed to evaluate the overall survival. The Wilcox test was carried out for comparisons between the two groups, and the Kruskal-Wallis test was used for comparisons of more than two groups. *p* < 0.05 represented statistical significance.

## 3. Results

### 3.1. Visualization of Mutation Profiling in Cutaneous Melanoma

Mutation profiling of cutaneous melanoma was analyzed and visualized using the maftools package. The frequency distribution and the statistics of different mutation types identified are summarized in Figure 1(a), in which the missense mutation was the most common mutation in the variant classification. Single nucleotide polymorphism (SNP) was the main variant type identified, and the C>T transition was the most frequently observed in single nucleotide variant (SNV) classification. In addition, the number of mutated bases for each patient was calculated, and mutation types were represented graphically using boxplots with different colors. Furthermore, the top 10 mutated genes were ranked in descending order according to the mutation frequency, and TTN accounted for the most common mutated gene. Moreover, a waterfall plot was depicted to display detailed mutation information relative to the top 30 significantly expressed genes in cutaneous melanoma patients (Figure 1(b)).

### 3.2. TMB and Clinical Correlation

The TMB value for each patient was calculated, and patients were classified into low and high TMB groups using the median of TMB value as the threshold. The Kaplan-Meier analysis was applied to evaluate the survival probability in different groups. As a result, the patients in the high TMB group presented a higher survival rate, indicating that higher TMB in cutaneous melanoma contributed to a better prognosis (Figure 2(a)). Moreover, we compared the relationship between the TMB level and clinical features in cutaneous melanoma. The results showed that TMB was associated with age (Figure 2(b)), sex (Figure 2(c)), and TN stage (Figures 2(d) and 2(e)). The TMB level was higher in males and patients over 65 years while it was lower in patients with advanced TN stage. Taken together, these results revealed that a higher TMB contributed to a better prognosis in cutaneous melanoma.

### 3.3. Identification and Functional Analysis of DEGs

In order to identify TMB-associated DEGs in cutaneous melanoma, an analysis using the DEG-seq2 R package was conducted. As shown in Figure 3(a), a total of 403 DEGs with ∣log2FC | >2 and FDR < 0.05, including 71 upregulated and 332 downregulated genes were identified. The GO enrichment analysis in Figures 3(b) and 3(c) indicated that DEGs were mainly implicated in epidermis development and skin development. In addition, the GSEA results revealed that DEGs participated in cancer-related pathways such as the cell cycle and DNA replication, as well as in immune-associated crosstalk including allograft rejection, graft-versus-host disease, and primary immunodeficiency (Figure 3(d)).

### 3.4. Identification of a TMB-Associated Signature

To identify whether DEGs may be responsible for the clinical prognosis, univariate COX regression and Kaplan-Meier survival analysis was conducted, and 91 DEGs were extracted for further analysis (Figure 4(a)). Subsequently, the Lasso COX regression and multivariate COX regression analysis were performed for the construction of a prognostic model (Figures 4(b) and 4(c)). Eight genes including TGM3, PROKR1, CRABP2, CHI3L1, PAEP, KLRK1, SLC32A1, and SPRR2F comprised the TMB-associated signature. The calculation of risk scores for each patient was based on the coefficients of each respective signature presented in Table 1. In addition, the patients were divided into the low- and high-risk groups according to the median of each risk score. The distribution of risk for patients and expression pattern of the eight prognostic genes are presented in Figure 4(d). The Kaplan-Meier analysis in the two groups demonstrated that patients with lower risk scores displayed better prognosis (Figure 4(e)).

### 3.5. Survival Probability Prediction

As shown in Figures 5(a) and 5(b), the results obtained from univariate and multivariate Cox proportional hazard model regression indicated that the TN stage and the risk scores of the TMB-related signatures were independent prognostic factors for cutaneous melanoma. The ROC curve analysis was performed to assess the predictive accuracy of the TMB-related prognostic model. The AUCs responsible for the 1-, 3-, and 5-year OS were 0.705, 0.726, and 0.7272, respectively (Figure 5(c)). In addition, a nomogram including age, sex, TMN stage, and the risk scores was constructed to predict OS at 3 and 5 years for cutaneous melanoma patients (Figure 5(d)).

### 3.6. Correlation between the Mutation Types of the Eight Prognostic Genes and Immune Infiltrates

We further investigated the correlation between the mutation types of the eight prognostic genes and the immune infiltrates of B cells, CD8+ T cells, CD4+ T cells, macrophages, neutrophils, and dendritic cells. Compared with the wild-type genes, infiltrations associated with mutations in the eight prognostic genes displayed lower levels of immune infiltrates (Figure 6).

### 3.7. Different Immune Cell Fractions in the Low- and High-Risk Groups

According to the CIBERSORT algorithm, we calculated the fraction of 22 immune cells present in each sample of cutaneous melanoma. In addition, the proportion of immune cells for different risk groups was compared using the Wilcox test and was then visualized using violin plots. As a result, the infiltration levels of plasma cells, CD8+ T cells, CD4+ memory activated cells, NK activated cells, and M1 macrophages were higher in the low-risk group than that in the high-risk group, while the infiltration of M0 macrophages, M2 macrophages, and activated dendritic cells was higher in the high-risk group (Figure 7).

## 4. Discussion

To date, immunotherapy is considered an attractive approach for tumor treatment. In recent years, with the availability of ICI therapy, the survival rate of patients with cutaneous melanoma has considerably improved. However, not all patients have benefited from such therapy, and the treatment effects vary from person to person, resulting in a substantial waste of healthcare resources and a heavy economic burden for patients. Hence, it is urgent to investigate novel effective immunotherapeutic targets to achieve the most benefit for patients.

Tumorigenesis is an intricate process, which involves mutations of multiple genes and a complicated interaction with the microenvironment. The occurrence of nonsynonymous mutations in tumor cells may generate new antigens, which are recognized by the autoimmune system and resulted in the activation of T lymphocytes and the immune response [20, 27, 28]. The greater the presence of new antigens, the more likely these will be recognized by the immune system, indicating the crucially significant role of TMB in ICI therapy. Studies have demonstrated that the TMB is closely correlated with the clinical prognosis of patients [29, 30]. In colorectal cancer, patients with high TMB had better prognosis when receiving combination therapy [31]. In the CheckMate 026 Investigators trial, patients with high TMB benefited from the treatment of nivolumab, while no effect was observed in the subgroup stratified by the PD-L1 expression [22], indicating the potential of TMB as a biomarker of immunotherapy outcome. A subsequent study research further confirmed the significant role of TMB, in which the investigators found that patients with high-TMB were closely associated with an enhanced response to nivolumab plus ipilimumab immunotherapy [32]. Jiang et al. demonstrated that a low TMB and high immune infiltrates of CD8+ T cells were predictive factors for longer survival in lung squamous cell carcinoma patients [33]. Moreover, in a study investigating diverse cancer types, the TMB was identified as an independent factor for predicting response to immune treatment [34]. Consistent with these studies, our findings showed that cutaneous melanoma patients having a higher TMB also had a higher survival rate than patients with a lower TMB. In addition, we also demonstrated that TMB was negatively associated with the stage of TN classification, which suggested that high TMB in cutaneous melanoma was a predictive factor of a better outcome.

Subsequently, the functional analysis of TMB-related DEGs revealed that the identified DEGs were implicated in the development of the epidermis and skin, as well as in immune-associated crosstalk such as allograft rejection, graft-versus-host disease, and primary immunodeficiency. Furthermore, a prognostic model consisted of TMB-related genes including TGM3, PROKR1, CRABP2, CHI3L1, PAEP, KLRK1, SLC32A1, and SPRR2F was established via the Lasso COX regression and multivariate COX regression analysis. Patients with high-risk scores presented poor prognosis, and the prognostic model displayed superior predictive accuracy evidenced by AUC of ROC analysis. Combined with the results of the proportional hazards model conducted by the multivariate Cox regression, our results strongly indicated that the model could act as an independent prognostic biomarker for cutaneous melanoma. Significantly, our results revealed that the expression of TMB-related signatures was related to the infiltration of different immune cells. The mutation of an eight gene TMB signature was associated with the inhibition of immune infiltration. Besides, our results found that the infiltration level of CD8+ T cells, CD4+ T cells, and NK-activated cells, as well as M1 macrophages, increased in the low-risk group. T lymphocytes are recognized to play a significant role in the antitumor immune response, and previous studies have demonstrated that T lymphocyte infiltrates closely correlated with better survival outcomes. In the studies of melanoma, patients with a higher degree of CD4+ tumor-infiltrating lymphocytes tend to have more favorable outcome [35]. Similarly, a positive association between infiltrating CD8+ lymphocytes and patient survival was observed in Piras's research [36]. Li et al. found that CD4+ T cells could stimulate the activation of M1 macrophages, and the infiltrate level of CD4+ and CD8+ T cells was negatively associated with tumor size in gastric cancer [37]. Furthermore, Mukhtar documented that the different subtype conversion of macrophages was crucial for tumor therapy as the M1 macrophages exerted antitumor activity via inducing adaptive immune responses, while M2 macrophages promoted tumor progression [38]. In accordance with the above studies, our findings showed that the infiltration of M0 and M2 macrophages was higher in the high-risk group than in the low-risk group, suggesting the significant role of macrophages in immune infiltration.

To our acknowledge, our investigation is the first study to develop a TMB-related prognostic model for the prediction of prognosis and to illustrate its potential association with immune infiltration in patients with cutaneous melanoma. Our study not only revealed the important role of TMB in survival outcome in cutaneous melanoma but also proposed a prognostic model for survival prediction, supplying new potential targets for immunotherapy. Nonetheless, several limitations need to be considered in our study. For example, an additional independent clinical cohort is required to validate the efficiency of the prognostic model, and further experimental studies are essential to further establish the biological role of the identified biomarkers.

In conclusion, our study provides evidence supporting the importance of TMB as a significant determinant of immunogenicity, and immune cell infiltration reflects the functional activity of the immune response. Our study elucidated the relationship between TMB-related signatures and immune infiltration, proposing that a prognostic model that includes TMB could represent a reliable predictor for predicting the efficiency of immunotherapy.

## Figures and Tables

**Figure 1:** Visualization of mutation profiling in cutaneous melanoma samples. (a) Frequency distribution and summary statistics of different mutation types. (b) Waterfall plot of mutation profiles in cutaneous melanoma samples. The top 30 genes with different mutation types are listed in order of mutation frequency. The different colors of the water plot represent different mutation types, which are annotated at the bottom. The bar plot on the right means the mutation frequency of each gene, while the above one represents the number of mutation burden.

**Figure 2:** The Kaplan-Meier analysis of TMB and the relationship with clinical risk characteristics. (a) The Kaplan-Meier analysis of patients with low- and high- TMB groups. (b–e) Statistically significant differences (*p* < 0.5) in patients stratified by age, sex, and T and N stages were evidenced by the Wilcox test. TMB: tumor mutation burden.

**Figure 3:** Identification and functional enrichment analysis of DEGs between the low- and high-TMB groups. (a) The volcano plot of DEGs (∣log(FC) > 2∣, FDR < 0.05). The upregulated DEGs were depicted in red, while the downregulated were in green. (b, c) GO enrichment analysis, including BP, CC, and MF, of DEGs. (d) Summary of GSEA results with *p* < 0.05. BP: biological process; CC: cell composition; MF: molecular function; GSEA: gene set enrichment analysis; TMB: tumor mutation burden.

**Figure 4:** Construction and assessment of TMB-related signature for cutaneous melanoma. (a) Visualization of the intersection of DEGs related to prognosis. (b, c) TMB-related genes associated with prognosis are identified by the LASSO COX regression. (d) Distribution of patients' status and TMB-related genes in the low- and high-risk groups. (e) The Kaplan-Meier analysis of patients in the low- and high-risk groups. TMB: tumor mutation burden.

**Figure 5:** Risk score is an independent prognostic factor for survival probability prediction. Univariate COX (a) and multivariate COX (b) regression analysis of clinical risk characteristics and risk score. (c) The ROC curves of TMB-related signature for 1, 3, and 5 years. (d) Construction of nomogram for predicting the OS probability of patients with cutaneous melanoma. TMB: tumor mutation burden; OS: overall survival; ROC: receiver operating characteristic.

**Figure 6:** The relationship between mutants of 8 prognostic genes and immune cells. (a–h) Comparisons of immune cell infiltration in different mutation types of 8 prognostic genes. ^∗^*p* < 0.05, ^∗∗^*p* < 0.01, ^∗∗∗^*p* < 0.001.

**Figure 7:** Comparison of different immune cell fractions in patients of low- and high- risk score. The low-risk group is colored green, while the high-risk group is colored red.

**Table 1:** Multi-Cox regression analysis of TMB-related signatures.

Id	Coef	HR	HR.95 L	HR.95H	*p* value
TGM3	0.01287	1.012953	0.999133	1.026965	0.066331
PROKR1	0.436863	1.547844	1.276414	1.876993	8.96E-06
CRABP2	0.001434	1.001435	0.999676	1.003197	0.109893
CHI3L1	-0.00265	0.997357	0.994393	1.00033	0.081346
PAEP	0.000235	1.000235	1.000113	1.000358	0.000156
KLRK1	-0.73979	0.477212	0.291349	0.781645	0.003298
SLC32A1	-15.5098	1.84E-07	4.41E-14	0.766073	0.046127
SPRR2F	0.036618	1.037297	1.01223	1.062985	0.003347

## Data Availability

The data can be downloaded from the TCGA database (https://portal.gdc.cancer.gov).
